# Leakage Current Sensor and Neural Network for  MOA Monitoring

**DOI:** 10.1155/2022/6728900

**Published:** 2022-06-17

**Authors:** Tao He, Yang Li, Zhong Zhang, Pengfei Shen, Yu Zhang

**Affiliations:** Ma'anshan Electric Power Supply Company, State Grid Anhui Electric Power Co Ltd, Ma'anshan 243000, China

## Abstract

Metal-oxide arrester (MOA) has been widely used in electric power systems. The leakage current monitoring of MOA can not only detect the MOA's running state continuously and intelligently but also reduce the unexpected outage of the equipment, which is also beneficial to the stability of the grid. The MOA loses its protection function due to various faults caused by excessive leakage current in actual running. This article studies the monitoring method of MOA based on leakage current sensor and back propagation (BP) neural network. At first, we design a novel leakage current sensor to acquire the leakage current of MOA. Then, the leakage current measurement of MOA based on harmonic analysis is proposed. Finally, the strong training ability of the BP neural network is used to train some key parameters that can reflect the aging of MOA so as to monitor the MOA state. The experimental results show that the leakage current acquired from the simulation is close to the actual leakage current that needs to be measured. It is also shown that the proposed method has good anti-interference and can effectively monitor the aging of MOA. Through the training of the BP neural network, the experiments prove that the training method in this article is superior to other neural network training methods obviously.

## 1. Introduction

The safety and stability of the electric power system have been involved with the rapid advance of the economy. It can be said that electrical equipment is important in society today. The world is committed to the development of the electric power system. The long-term stable running of the electric power system cannot be separated from the normal operation of such equipment. As a protective device to avoid the influence of high voltage, such as lightning strike, the MOA is close to the insulation state under the normal running of the electric power system [1, 2]. When the electric power system is overvoltage, the equivalent resistance of MOA decreases rapidly, and the leakage current flowing through the MOA increases instantly, which ensures that the MOA is broken down before the protected equipment so as to effectively suppress the overvoltage.

The main reason for the faults of MOA is that the valve plate is damp or aged. The dampness of the valve plate of MOA is mainly caused by some objective factors [3]. Moisture slowly seeps into the MOA and makes it damp for a long time running. Therefore, the poor housed MOA is one of the main reasons for its dampness [4]. The aging of the valve plate will be very different due to the uniformity being relatively poor. In this way, the potential distribution of the valve plate of MOA will have slowly deviated. Eventually, parts of the valve plates will deteriorate first, then the leakage current and power consumption of MOA will increase for a long time running. Another reason for the accelerated aging of the valve plate of MOA is that the running voltage loaded to both ends of the MOA is lower than the normal voltage. When the MOA is running, especially single line-to-ground, the loaded voltage of the MOA is increased, which results in the fast aging of the valve plate of the MOA. Therefore, in order to detect the drawbacks of the MOA in time and avoid the accidents caused by the leakage current of MOA, we need to monitor and evaluate the running state of the MOA frequently to ensure the safe and stable running of the electric power system.

Accordingly, the main contributions of this article are summarized as follows. (i) We design a novel leakage current sensor to acquire the leakage current of MOA. (ii) The leakage current measurement of MOA based on harmonic analysis is proposed. (iii) BP neural network is used to train some key parameters that can reflect the aging of MOA.

The remaining of this article is organized as follows.  Section 2 reviews the related work. In Section 3, we study the acquirement and measurement of MOA leakage current. In Section 4, we propose the monitoring method of MOA based on the BP neural network. The experimental results are shown in Section 5.  Section 6 concludes this article.

## 2. Related Work

The first important step for monitoring MOA is the current measurement using a sensor. The current sensor is an important current measurement product, which measures the magnetic field indirect current generated by the primary current. After signal processing, the current sensor outputs a low voltage or low current signal. There have been many sensors studied for current measurement. In [5], a quasidigital flux gate sensor was designed based on the duty-ratio model, and the mathematical model between the excitation voltage period and the measured current, which exceeded the measurement range, was built by analyzing the working principles of the duty-ratio model digital sensor. In [6], the authors presented an innovative common-mode current sensor node for the insulation monitoring framework of power distribution systems based on magnetic field analysis. In [7], the authors proposed an advanced current sensor with a dual-core topology based on differential-mode measurement. An analytical model of the magnetic field of the dual-core sensor was originally presented, which helped clarify the significance of the inner core in filtering noises and reducing the influence of system operation and cable positioning. In [8], the authors described a high-current sensor operating in a range up to 100 and 7.7 kA resolution. The system consisted of a self-integrating Rogowski coil connected to the electret sensor by a coaxial cable. In [9], the authors presented the design, fabrication, and characterization of two compact fiber-optic current sensors based on fiber Bragg gratings and the magnetostrictive alloy Terfenol-D.

Many strategies of third-harmonic measurement have been proposed. In [10], the authors presented the solution of the third-harmonic generator model used for a stator-ground fault study in terms of the mesh currents and used the derived equations to develop a third-harmonic based fault location method. In [11], the authors proposed a method to estimate all electrical parameters of five-phase induction motors based on a new concept of instantaneous impedance. In [12], the authors performed power-dependent third-harmonic generation measurements on gated single-layer graphene and detected a significant deviation from the cubic power law expected for a third-harmonic generation process. In [13], the authors discussed the effects of third-harmonic current injection on a five-phase permanent magnet synchronous machines with a conventional magnet shape depending on the saturation. In [14], the authors presented the first experimental validation of the stability analysis based on the online measurement of harmonic impedances exploiting the linear time-periodic approach applied to ac networks of power converters. In [15], the authors proposed an online monitoring technique for the surge arrester under dry and pollution conditions when measuring either the total leakage current or both the internal and external leakage currents of three different types of surge arresters. In [16], the authors designed a circuit measuring resistive current based on leakage current standard waveform of the surge arrester. In [17], the authors proposed the development of load signatures by a limited number of harmonic current vectors. In [18], the authors presented a harmonic model for metal-oxide surge arresters that could be utilized to simulate their performances under applied harmonic voltage. In [19], the authors proposed a newly developed technique, referred to as a hybrid method, to extract resistive leakage current without acquiring the grid's voltage. In [20], a new current decomposition method based on multiple linear regression was presented. The time-domain equations of every current component on the applied voltage were deduced based on an improved equivalent model of the MOA arrester.

Currently, there are many training methods for the monitoring of MOA. In [21], a Kohonen neural network was proposed for the MOA fault diagnosis. For the problem of online monitoring parameters of MOA, that is, suffering from the external environment interference in the power system, in [22], a novel MOA parameters modified method by eliminating external environmental factors interference was proposed.

In recent times, there have been a lot of studies on the current sensor and third-harmonic leakage current, but the neural network is seldom used to monitor the running state of MOA. Based on this, we study the monitoring method of MOA based on leakage current sensor and neural network.

## 3. The Leakage Current Acquirement and Measurement of MOA

### 3.1. A Novel Leakage Current Sensor

The acquisition of leakage current is a key step in MOA monitoring. The leakage current only with mA-level of MOA is very small under normal voltage. The interference is very strong in the acquisition process, so the leakage current extraction is very important. The leakage current acquisition methods include direct coupling (end shield disconnection) and magnetic coupling (cross-core sensor). The current acquisition accuracy of direct coupling is relatively high, but it is rarely used now because the related running is unfavorable for the safety and stability of the electric power system, while the magnetic coupling is used much more in practice. According to the characteristics of MOA, we propose a resistance sensing method to acquire the leakage current of MOA without peeling the end shield so that there is no effect on the high-side voltage. The lower end of MOA is connected with counters that record MOA running times, and its resistance is usually hundreds of ohms. The leakage current can be inferred from detecting the pressure drop of the leakage current on MOA. There is a relationship between counterresistance and counterparameters, and the value of counterresistance is not constant, so it must be monitored.

Let *R*_*1*_*, R*_*2*_,…, *R*_*n*_ be the resistance used for measurement in monitoring. Since the resistance *R*_*c*_ and *R*_*1*_*, R*_*2*_,…, *R*_*n*_ of the counter are far less than the resistance value of MOA (usually above MΩ), the influence of *R*_*1*_*, R*_*2*_,…, *R*_*n*_ on the leakage current *I*_*lc*_ of MOA can be ignored. The resistance value *R*_*c*_ is too high, which leads to the fault of the counter, and it will also affect the detection. *R*_*1*_ is usually connected to both ends of the counter in parallel first, and the voltage of *R*_*1*_ is measured as *U*_*1*_. Similarly, the voltage measured after parallel connection of *R*_*n*_ through relays is *U*_*n*_. The number of parallel connections depends on the required accuracy. A novel leakage current sensor designed in this article can calculate *R*_*c*_ by connecting two resistances in parallel but can calculate the resistance value of multiple counters by connecting more resistances, which makes the errors decline. The leakage current *I*_*lc*_ and the resistance value of the counter *R*_*c*_ are defined as follows:

(1) $$\begin{array}{c} I_{lc}=\left(\frac{1}{R_{i}}+\frac{1}{R_{c}}\right)\times U_{i}=\left(\frac{1}{R_{i}}+R_{j}+R_{c}\right)\times U_{j}, \end{array}$$

(2) $$\begin{array}{c} R_{c}=\frac{R_{i}R_{j}\times \left(U_{i}-U_{j}\right)}{\left[R_{i}\times U_{j}-R_{j}\times \left(U_{i}-U_{j}\right)\right]}. \end{array}$$

After the counterresistance is calculated, the leakage current *I*_*lc*_ of MOA can be acquired by measuring the voltage at both ends of MOA with equation (1) and equation (2). As a result, the leakage current is calculated by the pressure drop between the sampling resistances and the counterresistance. There is a high demand for accuracy and stability for sampling resistances *R*_*1*_, *R*_*2*_,…, *R*_*n*_, so we use standard resistance with minimal temperature drift which can completely remove the phase-shifted current in the magnetic ring sensor measurement.

### 3.2. The Leakage Current Measurement of MOA Based on Harmonic Analysis

The internal MOA can be equivalent to a parallel circuit with good nonlinear resistance and surface-to-ground capacitance. Therefore, the leakage current is resistive-capacitive, and the resistive current only accounts for 10%–20%. Because of the nonlinear characteristics of the valve plate of MOA, there are a lot of high harmonic components in the resistive leakage current. During the long-term running of MOA, the main reason for the decline of its insulation performance is the internal moisture and aging of the valve plate, which is mainly reflected in the significant increase of resistive fundamental current and resistive third-harmonic components of MOA under normal working voltage, while its capacitive current components are relatively stable. At present, the monitoring method of MOA is usually used to detect the running state of the MOA, which has been put into running by monitoring the change of the leakage current so as to detect the fault of MOA in time. The common leakage current measurement methods of MOA include the capacitive current compensation method, fundamental wave method, and third-harmonic method.

The new method of leakage current harmonic analysis is based on compensation technology, which eliminates the influence of the third-harmonic current components caused by the harmonic voltage of the electric power system on the leakage current measurement so that the third-harmonic current components can be acquired by MOA alone. Moreover, the relationship between the resistive third-harmonic current and the total resistive current is established. The circuit of MOA and sensor is shown in Figure 1.

Let *I*_*h*_^(*k*)^ denote the *k*th harmonic of the current *I* and the third-harmonic of the voltage produces a capacitive current component with the same frequency, which contributes greatly to the total third-harmonic current *I*_*t*_^(3)^. However, the total third-harmonic current *I*_*t*_^(3)^ minus capacitive third-harmonic current *I*_*c*_^(3)^ and then the resistive third-harmonic current *I*_*rh*_^(3)^ are generated by the MOA nonlinear resistance:

(3) $$\begin{array}{c} I_{rh}^{\left(3\right)}=I_{t}^{\left(3\right)}-I_{c}^{\left(3\right)}. \end{array}$$

On the one hand, *I*_*rh*_^(3)^ refers to the resistive third-harmonic current. The amplitude and phase angle of the current *I*_*t*_^(3)^ are measured by the total leakage current *I*_*t*_ at the grounding terminal of the MOA. On the other hand, *I*_*c*_^(3)^ can be indirectly determined through the measurement of the electric field.

#### 3.2.1. Capacitive Harmonic Current

The capacitive third-harmonic current *I*_*c*_^(3)^ can be determined by measuring the probe current *I*_*p*_ located in the MOA electric field, and the third-harmonic probe current *I*_*p*_^(3)^ can be acquired by the Fourier transform of *I*_*p*_. If the amplitude and phase angle of are related to *I*_*c*_^(3)^, the resistive third-harmonic current *I*_*rh*_^(3)^ can be acquired according to equation (3). *I*_*c*_^(3)^ mainly depends on the third-harmonic voltage of the phase where the MOA is located. To some extent, the influence of stray capacitance is also related to the voltage of the adjacent phase, while the probe current *I*_*p*_^(3)^ is only related to the stray capacitance, which indicates that *I*_*p*_^(3)^ is more affected by the adjacent phase.

It is reasonable to assume that the third harmonic of the phase voltage has the same phase angle as the fundamental frequency of each phase, if only the fundamental frequency and third harmonic are considered, which can be defined as follows:

(4) $$\begin{array}{c} U_{h}^{\left(k\right)}=\ln\cos\left(2\pi fft+\frac{2n\pi }{3}\right)+U_{h}^{\left(3\right)}\cos\left(3\times 2\pi fft+2\pi n\right), \end{array}$$

where *n* = 0, 1, and 2 express three phases and *f* is the fundamental frequency.

It can be seen from equation (4) that the main advantage of the leakage current third-harmonic analysis is that the phase angle difference of all the third-harmonic voltage *U*_*h*_^(3)^ is a multiple of 2*π*. Therefore, *U*_*h*_^(3)^ can be regarded as the zero-sequence voltage with three times the frequency of the fundamental frequency of the system. Accordingly, *I*_*p*_^(3)^ and *I*_*c*_^(3)^ have the same phase angle, which are unrelated to the position of the field probe.

A calibration process for *I*_*p*_^(3)^ must be introduced before the amplitude of *I*_*c*_^(3)^ can be determined because the capacitance of the field probe is usually unknown. The calibration is based on a comparison of the fundamental frequency components *I*_*t*_^(1)^ and *I*_*p*_^(1)^. Since *I*_*t*_^(1)^ is mainly capacitive and its amplitude is not sensitive to the growth of the resistive current components, so it can be considered reasonable. The fundamental current increases by only a few percentages over the actual range of resistive current. Therefore, in fact, *I*_*t*_^(1)^ can be considered as equal to *I*_*c*_^(1)^, and the relationship between the amplitude of fundamental frequency components *I*_*t*_^(1)^ and *I*_*p*_^(1)^ can be defined as follows:

(5) $$\begin{array}{c} AMP_{1}=\frac{I_{t}^{\left(1\right)}}{I_{p}^{\left(1\right)}}. \end{array}$$

According to equation (6), the capacitive third-harmonic current can be determined as follows:

(6) $$\begin{array}{c} I_{c}^{\left(3\right)}=AMP_{3}\times I_{p}^{\left(3\right)}. \end{array}$$

Generally, AMP_3_ is not equal to AMP_1_, so AMP_3_ needs to be introduced. According to equation (5) and equation (6), assuming that *I*_*t*_^(1)^ is equal to *I*_*c*_^(1)^, then *I*_*c*_^(1)^ can be defined as follows:

(7) $$\begin{array}{c} AMP_{3}=\frac{AMP_{1}\cdot I_{p}^{\left(3\right)}}{I_{b}^{\left(3\right)}}\times \frac{I_{c}^{\left(3\right)}}{I_{p}^{\left(3\right)}}. \end{array}$$

For each frequency, the current is proportional to the field strength, so equation (7) can also be expressed as follows:

(8) $$\begin{array}{c} AMP_{3}=\frac{AMP_{1}\cdot E_{p}^{\left(1\right)}}{E_{p}^{\left(1\right)}}\times \frac{E_{c}^{\left(3\right)}}{E_{p}^{\left(3\right)}}. \end{array}$$

The relationship between the fundamental frequency and the electric field components of the third-harmonic is constant and irrelevant to its spatial position in single-phase application, which means that AMP_3_ and AMP_1_ are equal. As discussed above, there is a corresponding phase shift for the third-harmonic components, so that AMP_3_ and AMP_1_ are not equal in three-phase applications in general.

#### 3.2.2. The Calculation of Electric Field

In order to determine the relationship between AMP_3_ and AMP_1_ at the field probe, the field strength of two typical three-phase MOA at their base is calculated. The field strength is calculated at two system voltages, which are 145 kV (single-phase MOA) and 420 kV (three-phase MOA), with a wide range of phase spacing.

Table 1 shows the structure of MOA. Assuming that the MOA is adjacent to the wall, which simulates a large grounded object such as a transformer. We should notice that the effect of the wall on the electric field strength is small compared with that of the adjacent phase.

The electric field strength at the base of MOA is calculated by the boundary element method [23], which is developed for the three-phase application. The normal voltage of MOA for calculation is shown in Table 2.

Field strength *E*_*c*_^(1)^ and field strength *E*_*c*_^(3)^ are distributed at the base of MOA, while field probes *E*_*p*_^(1)^ and *E*_*p*_^(3)^ are located 10 cm below and 5 cm away from the base of MOA. The electric fields of the two types of MOA are given in the form of AMP_3_/AMP_1_ in Table 3. Although there are significant differences between MOA configurations such as phase spacing, single-phase, or three-phase, as can be seen from Table 3, AMP_3_/AMP_1_ is basically a constant. A single ratio of the single-phase or three-phase configuration can be used for all system voltage levels in real use.

#### 3.2.3. Determination of Resistive Third-Harmonic Leakage Current

According to equation (3), equation (5), and equation (6), the resistive third-harmonic leakage current of MOA can be determined from the following equation:

(9) $$\begin{array}{c} I_{rhl}^{\left(3\right)}=I_{t}^{\left(3\right)}-0.75\times \frac{I_{t}^{\left(1\right)}}{I_{p}^{\left(1\right)}}\times I_{p}^{\left(3\right)}. \end{array}$$

As mentioned above, the resistive third-harmonic leakage current can be used to determine the condition of MOA during running. However, it can only be limited to comparative measurement since we do not usually know the resistance third-harmonic current target value of MOA.

The accurate measurement of resistive current components in MOA leakage current plays an important role in monitoring the faults of MOA. The leakage current of the third harmonic of MOA is defined as follows. The resistive third-harmonic current *I*_*rh*_^(3)^=*εUα*, while *U* is the normal working voltage applied to both ends of MOA.

(10) $$\begin{array}{c} I_{hl}^{\left(3\right)}=\frac{U_{h}^{\left(3\right)}}{dt}+\varepsilon U_{h}^{\alpha }-I_{t}^{\left(3\right)}+0.75\times \frac{I_{t}^{\left(3\right)}}{I_{p}^{\left(3\right)}}\times I_{p}^{\left(3\right)}+\varphi_{3}, \end{array}$$

where *ε* and *α* are the coefficients determined by the nonlinear characteristics of MOA. *U*_*h*_^(*n*)^ is the amplitude of harmonic voltage and *φ*_*n*_ is the phase of harmonic voltage.

## 4. The Monitoring of MOA Based on BP Neural Network

MOA directly withstands the effect of electric power system operating voltage for a long time without externally gapped line arrester. It is probably not housed well due to the poor structure of MOA, which makes the resistance plate easy to be affected by moisture in running. When the resistance plate is affected by moisture, the leakage current increases and the deterioration will be aggravated; thereby, the leakage current increases further.

The resistive current components of the leakage current increase the temperature of the resistance plate, resulting in wattful loss, which will also lead to MOA damage or explosion in severe cases, and then a large area of a power outage is generated. As MOA is an important device to limit the overvoltage of electric power systems, it is particularly important to monitor the performance of MOA in running to ensure the safe and stable operation of the grid. In this article, the BP neural network is used to train some key parameters, which can reflect the aging condition of MOA, so as to monitor the MOA state.

### 4.1. BP Neural Network

The neural network is widely used in pattern recognition, control optimization, intelligent information processing, and fault diagnosis because of its characteristics of distributed parallel processing, nonlinear mapping, adaptive learning, and robust-fault tolerance. Currently, BP neural network is the most widely used prediction model [24]. The weight and threshold of the BP neural network are usually adjusted along the negative gradient direction of the network error change, and finally, the network error reaches the minimum. There are three layers in BP neural network, including input layer, hidden layer, and output layer.

The common fault types and fault causes during MOA running are shown in Table 4 [25, 26], where 0 indicates that the phenomenon does not happen and 1 indicates that the phenomenon happens.

In Table 4, I is the critical operating voltage U_1mA_ at 1 mA direct current with a change of more than ±5% or the leakage current greater than 50 *μ*A under 0.75 U_1mA_. II is the doubling of the resistance current. III is the increasing of alternating current leakage current under operating voltage. IV is the insulation resistance lower than 1000 MΩ. V is the surface flashover. VI is an explosion. VII is raising temperature. Fault type 1 is the resistance plate with moisture; 2 is the initial aging; 3 is the surface pollution; 4 is the poor fastening of the terminal; 5 is the aging of parallel resistance; 6 is the poor manufacturing quality of the resistance plate.

We use the newff() function to build a trainable BP neural network, which uses seven fault causes as its inputs and six fault types as its outputs. For the first sample, the input vector V1 = (1011010), and the expected output value *E*1 = (100000).

### 4.2. Training for BP Neural Network

The adaptive modified learning rate algorithm (traingda) is used as the learning algorithm. Traingda is a network training function that updates weight and bias values according to gradient descent with an adaptive learning rate. The initial value of the learning rate is 0.85. The learning rate descent factor and the learning rate ascent factor are taken as the default values. The number of training time is 50. The momentum factor is 0.9. The maximum number of iterations is l000. The learning objective is 0.00001.

It is assumed that an input vector (0100101) is acquired through a novel leakage current sensor and the resistive third-harmonic leakage current measurement method designed in this article, and then it is input into the BP neural network. The output is the membership degree of the fault cause relative to each fault.

The following uses the fuzzy information processing-related theory to verify the accuracy of the BP neural network. Let the fault domain *d* = (*P1, P2*, ..., *P*7) constitute fuzzy power set *F*(*d*). For any fault *A* ∈ *F*(*d*), the relative Euclidian distance of fault A to six typical faults can be defined as follows:

(11) $$\begin{array}{c} re_{m}\left(P\right)=\sqrt{\frac{1}{7}{\sum_{n=1}^{7}\left(P_{n}-P_{m}\right)}^{2}},\;m=1,2,\ldots ,6. \end{array}$$

In equation (11), *m* is set from one to six according to reference [27]. In order to compare the membership function *mf*_*m*_(*P*)=cos  *re*_*m*_(*P*), according to the maximum membership degree principle, the fault of MOA can be acquired, which is similarly to the bias balanced by the orthogonal design decision mechanism [28], and the results are shown in Table 5.

As can be seen from Table 5, when the threshold is 0.1, BP neural network diagnoses the MOA fault as No. 2 (initial aging) and No. 4 (poor fastening of the terminal). The conclusion is in accordance with the diagnostic conclusion when the threshold value is 0.8 in the membership function.

## 5. Experiment and Results Analysis

### 5.1. Leakage Current Measurement

In order to verify that the MOA leakage current measurement based on the third harmonic proposed in this article has a good anti-interference performance to harmonic voltage. We use MATLAB to simulate the voltage containing harmonic voltage. The steps are summarized as follows:

**Step 1 .**

Simulating the operating voltage with different harmonic voltage and replacing the operating voltage applied at both ends of MOA in real.

**Step 2 .**

Setting the initial value (*α*, *ε*, *c*) of equation (10). Taking the calculated leakage current as the actual leakage current. In this article, *α* = 15, *ε* = 0.1, and *c* = 10^−10^ pF.

**Step 3 .**

The calculated leakage current is fitted to approximate the actually measured leakage current.

According to the simulation of different harmonic voltages in Step 1, we propose four operating voltages with different harmonics.

**Case 1 .**

*U*_*h*_^(3)^  = 0.

**Case 2 .**

*U*_*h*_^(3)^  = 2%, *φ*_*3*_ = 0°.

**Case 3 .**

*U*_*h*_^(3)^  = 3%, *φ*_*3*_ = 90°.

**Case 4 .**

*U*_*h*_^(3)^  = 5%, *φ*_*3*_ = 180°.

In the above four different cases, *U*_*h*_^(*n*)^ is the amplitude of harmonic voltage and *φ*_*n*_ is the initial phase of harmonic voltage.

We use equation (10) to calculate the leakage current as the actual measured leakage current, and the leakage current calculated by the method proposed in this article is fitted with the actual measured leakage current. The measurement results under four different cases are shown in Figure 2.

As seen from Figure 2, there are harmonics in the current that the leakage current *I* actually measured and the leakage current *I*_*l*_ calculated are almost coincide. The method with high stability used in this article is almost little affected by harmonic voltage content and initial phase in the grid so that it can eliminate the influence of harmonics on the leakage current measurement. In addition, it also can be seen from Figure 2 that the resistive harmonic current *I*_*rh*_ will increase with the voltage harmonic content increasing, which indicates that the harmonic content of operating voltage is an important factor in promoting the aging of MOA. The proposed method has good anti-interference to harmonic voltage content and the initial phase of grid voltage, and it also can be applied to MOA monitoring.

### 5.2. Comparison Analysis

Evaluation indicators in BP neural network-based MOA monitoring method include precision ratio (P), recall ratio (*R*), and *F*1. The purpose of the experiment is to verify that the BP neural network training used in the monitoring method of MOA is superior to other neural network training methods. We choose the guided anchoring method of faster region-based convolutional neural network (GA_Faster R–CNN) [29], yielding multifold training deep neural network (YMufT-DNN) [30], domain phrase attention-based hierarchical recurrent neural network (DPA-HNN) [31], and online monitoring method of MOA based on passive RFID (OM_MOA-pRFID) [2] for comparison.

The experimental results are shown in Table 6 and Figure 3.

It can be seen from Table 6 and Figure 3 that the proposed method in this article has good performance in *P*, *R*, and *F*1. The BP neural network can automatically extract reasonable solution rules by learning the instance set with correct answers; that is, it has the ability of self-learning. One of the most remarkable things about this experiment is that the *F*1 of YMufT-DNN and OM_MOA-pRFID is close to that of the proposed method in this article. It is because the OM_MOA-pRFID monitoring algorithm can accurately calculate the relevant parameters reflecting the state of MOA. Since the pooling layer of CNN loses a lot of valuable information and ignores the partial and whole correlations, the *P*, *R,* and *F*1 of GA_Faster R–CNN do not exceed 0.8.

In addition, the response time is a very important metric for the monitoring of MOA. In Figure 4, we compare the response time of the proposed method in this article with the other four baselines. It can be seen that the proposed method in this article required less total response time and training response time to train the monitoring of MOA than the other four baselines. Significantly, the YMufT-DNN has a good performance in training response time that the yielding multifold training (YMufT) strategy helps the deep neural network model to converge faster.

## 6. Conclusions

This article proposes the monitoring method of MOA based on leakage current sensor and BP neural network for the aging of MOA, which needs to be detected. We design a novel leakage current sensor to acquire the leakage current of MOA, and a new method of MOA leakage current measurement based on harmonic analysis is proposed, which eliminates the influence of third-harmonic current components caused by the harmonic voltage of the electric power system on the leakage current measurement. Then, we use BP neural network to train key parameters that can reflect the aging of MOA. The experimental results show that the proposed method in this article has good performance in monitoring the MOA state.

As the running state of MOA changes with time and working conditions, and the way of describing the fault types and fault causes after the fault varies considerably from person to person, the fault sets should be refined and supplemented in the future work in order to meet the needs of the project.

## Figures and Tables

**Figure 1:** The circuit of MOA and sensor.

**Figure 2:** Comparison of calculation results.

**Figure 3:** The comparison of training methods using neural network.

**Figure 4:** The comparison of response time.

**Table 1:** The structure of MOA.

Size	145 kV	420 kV
Phase spacing (m)	1.6	5.1
The height of MOA (m)	3.4	6.5
The distance from the wall (m)	1.2	3.1

**Table 2:** Normal voltage of electric field calculation.

Frequency components	Phase		
	1	2	3
Fundamental frequency	−50	100	−50
Third harmonic	100	100	100

**Table 3:** AMP_*3*_/AMP_1_.

Voltage (kV)	Phase		
	1	2	3
145	0.71	0.7	0.71
420	0.83	0.81	0.83

**Table 4:** Fault types and fault causes during MOA operation.

Fault type	Fault cause						
	I	II	III	IV	V	VI	VII
1	1	0	1	1	0	1	0
2	0	1	0	1	0	0	1
3	0	0	1	0	1	0	0
4	0	0	0	0	1	0	0
5	0	0	0	0	0	1	0
6	1	0	1	1	1	1	1

**Table 5:** MOA fault diagnosis result.

Fault no.	BP neural network diagnosis result	The membership degree
1	0.0000	0.5516
2	0.1728	0.9274
3	0.0001	0.7923
4	0.3536	0.8617
5	0.0005	0.6621
6	0.0395	0.6621

**Table 6:** The performance of neural network training.

	Precision ratio	Recall ratio	*F*1
GA_Faster R–CNN	0.701	0.727	0.713
YMufT-DNN	0.736	0.756	0.849
DPA-HNN	0.742	0.759	0.765
OM_MOA-pRFID	0.766	0.791	0.884
This article	0.822	0.838	0.898

## Data Availability

All data used to support the findings of the study are included within the article.
